The article "A Three-Dimensional Cement Quantification Method for Decision Prediction of Vertebral Recompression after Vertebroplasty" was retracted in 2023. Reasons: signs of a paper mill; suspected computer-generated content; unreliable results or conclusions; concerns about the data.

# A Three-Dimensional Cement Quantification Method for Decision Prediction of Vertebral Recompression after Vertebroplasty

**DOI:** 10.1155/2022/2330472

**Published:** 2022-05-12

**Authors:** Yanming Zhang, Tao Zhang, Xiang Ge, Yong Ma, Zhenduo Cui, Shuilin Wu, Yanqin Liang, Shengli Zhu, Zhaoyang Li

**Affiliations:** ^1^Tianjin Key Laboratory of Composite and Functional Materials, School of Materials Science and Engineering, Tianjin University, Tianjin 300350, China; ^2^Department of Orthopedic Surgery, Tianjin First Central Hospital, Tianjin 300190, China; ^3^Key Laboratory of Mechanism Theory and Equipment Design of Ministry of Education, School of Mechanical Engineering, Tianjin University, Tianjin 300354, China; ^4^Pain Department, The Third People's Hospital of Yunnan Province, Kunming 650010, China

## Abstract

**Objective:**

Proposing parameters to quantify cement distribution and increasing accuracy for decision prediction of vertebroplasty postoperative complication.

**Methods:**

Finite element analysis was used to biomechanically assess vertebral mechanics (*n* = 51) after percutaneous vertebroplasty (PVP) or kyphoplasty (PKP). The vertebral space was divided into 27 portions. The numbers of cement occupied portions and numbers of cement-endplate contact portions were defined as overall distribution number (oDN) and overall endplate contact number (oEP), respectively. And cement distribution was parametrized by oDN and oEP. The determination coefficients of vertebral mechanics and parameters (*R*^2^) can validate the correlation of proposed parameters with vertebral mechanics.

**Results:**

oDN and oEP were mainly correlated with failure load (*R*^2^ = 0.729) and stiffness (*R*^2^ = 0.684), respectively. oDN, oEP, failure load, and stiffness had obvious difference between the PVP group and the PKP group (*P* < 0.05). The regional endplate contact number in the front column is most correlated with vertebral stiffness (*R*^2^ = 0.59) among all regional parameters. Cement volume and volume fraction are not dominant factors of vertebral augmentation, and they are not suitable for postoperative fracture risk prediction.

**Conclusions:**

Proposed parameters with high correlation on vertebral mechanics are promising for clinical utility. The oDN and oEP can strongly affect augmented vertebral mechanics thus is suitable for postoperative fracture risk prediction. The parameters are beneficial for decision-making process of revision surgery necessity. Parametrized methods are also favorable for surgeon's preoperative planning. The methods can be inspirational for clinical image recognition development and auxiliary diagnosis.

## 1. Introduction

Osteoporosis compression vertebral fracture (OCVF) is a compression fracture of a single vertebral body or multiple vertebral bodies caused by a reduction in bone mineral density (BMD). It can lead to back pain, spinal deformity, decreased mobility in older people [1], and higher risk of age-adjusted mortality [2], all of which increase public health pressure. In most cases, percutaneous vertebroplasty (PVP) or kyphoplasty (PKP) is used to stabilize the wounded vertebrae to prevent further damage [3]. This kind of minimally invasive surgery improves the quality of life of patients with an OCVF by prompting pain reduction and mobility restoration [4]. Cemented vertebral failure can cause many complications, and research found that different cement distributions and volumetric factors greatly determine vertebral mechanical stability and appearance of complications [5]. The cement distribution can largely affect the prediction on risk of vertebral recompression and decisions on revision surgery of poorly augmented vertebrae.

The article "A Three-Dimensional Cement Quantification Method for Decision Prediction of Vertebral Recompression after Vertebroplasty" was retracted in 2023. Reasons: signs of a paper mill; suspected computer-generated content; unreliable results or conclusions; concerns about the data.

Volumetric factors were proposed to quantify the intravertebral cement distribution and evaluate the effect on vertebroplasty complications, such as intravertebral cement volume (CV), cement height in X-ray slices, cement morphology, and volume fraction [6–8]. Volume fraction (VF) is defined as the fraction of intravertebral cement volume to vertebral body volume and is meant to quantify the extent of cement filling given differences in vertebral size. Although these two risk factors can parametrically quantify the amount of cement, conflicting results on these factors have been presented in several studies [9, 10].

Research has shown that uneven mechanical support from the cement decreases the strength of augmented vertebrae [11, 12]. The compactness of cement is one of the risk factors that describes the cement distribution morphology, which is usually determined by X-ray or CT slices. In this case, the cement compactness was simply divided into lump and interdigitated types. The lump distribution pattern has been found to be a harmful distribution for augmented vertebrae. Since under this situation, the vertebrae are more easily to collapse again [6, 7]. Some clinical studies were conducted to parametrize cement morphology, suggesting that a more extensive and interdigitated distribution would increase the recuperative rate from OCVFs [8, 13, 14]. The obvious disadvantage of compactness factors is that two categories cannot parametrically parametrize the distribution cement. Also, the morphological information in two-dimension X-ray slices is difficult to replicate. Thus, the numerical relationship between three-dimensional cement distribution with vertebral mechanics remains unclear, and a new method for parametrizing the cement distribution is needed.

The article "A Three-Dimensional Cement Quantification Method for Decision Prediction of Vertebral Recompression after Vertebroplasty" was retracted in 2023. Reasons: signs of a paper mill; suspected computer-generated content; unreliable results or conclusions; concerns about the data.

Patient-specific multidetector computational tomography- (MDCT-) based finite element analysis (FEA) is a promising tool for assessing clinically relevant parameters. For vertebroplasty, some homogeneous FEA research has studied different injection volumes, cement modulus, cement-endplate contacts, and so on [15, 16]. For kyphoplasty, a study of the placement and symmetry of cement clouds [11], the author stated that the symmetric distribution of cement clouds is favorable. Several heterogeneous nonlinear FEA studies have been conducted to understand the mechanical effect of using various modulus of cement. A time-lapse microcomputed tomography (*μ*-CT) FEA study showed that the VF% was related to the stiffness gain percentage [17]. Chevalier et al. [15] found that different cement-endplate contact modes can dominate the stiffening and strengthening effects of augmentation. Excluding the research above, FEA studies focused on how cement morphology parametrically affects cemented vertebral mechanics are rare. On the other hand, it lacks a substantial quantification method to evaluate the augmentation. Parameters that correlate well with augmented vertebral mechanics are needed.

This study is aimed at investigating and parametrizing different cement distribution modes. Correlated well with failure risk of cemented vertebrae, these parameters can be utilized as efficient postoperative evaluating scales like other clinic postoperative risk factors, such as VAS score, kyphotic restoration, and vertebral height restoration. Thus, it should be used as reference on decision-making of early revision surgery. Patient-specific FEA testing was used to assess mechanical properties of cemented vertebrae. By dividing intravertebral space into 27 portions (cubes) according to vertebral anatomy, the cement morphology and distribution inside vertebrae were parametrized. Regression studies revealed parameters that correlated well with vertebral mechanics. Different types of cement were also evaluated in this study.

## 2. Materials and Methods

### 2.1. Data Collection

The MDCT datasets of patients with OCVF who underwent vertebroplasty were collected from local clinics between April 2017 and December 2020. Data collection was performed under the supervision of a clinical ethical committee, and all datasets were anonymized to protect privacy. The MDCT scans were taken by a Siemens Somatom Definition AS scanner (Siemens, Malvern, PA), with 120 kVp tube voltage, 210 mA current, 0.4 mm pixel size, and 1 mm slice thickness. The reconstruction kernel was set as the standard (B30S).

The article "A Three-Dimensional Cement Quantification Method for Decision Prediction of Vertebral Recompression after Vertebroplasty" was retracted in 2023. Reasons: signs of a paper mill; suspected computer-generated content; unreliable results or conclusions; concerns about the data.

The inclusion criteria for collection were as follows: (1) single or multiple vertebral levels between T10 and L4 in patients diagnosed with OCVFs who underwent PKP or PVP; (2) OVCFs without damaged vertebral posterior walls, nerve lesions, or intravertebral clefts (IVCs); and (3) clear visualization of cement cloud in digital imaging and communications in medicine (DICOM) sets. The exclusion criteria for collection were as follows: (1) severe cement leakage to the adjacent levels or spinal cord compression; (2) complete burst fracture at the cemented level due to its integrity that was not eligible for building a regular FEA model; and (3) vertebrae with posterior fixation constructs. A total of 51 vertebrae from 39 patients were eligible for inclusion and were investigated in the following study (Table 1).

### 2.2. Heterogeneous Finite Element Model Development

The workflow of model development is depicted in Figure 1. Briefly, MDCT data were imported into medical 3D reconstruction software Mimics (Materialise NV, Harislee, Belgium) to perform level segmentation and bone reconstruction, and masks of vertebrae and radiopaque bone cement were generated separately. The posterior ligamentous complex (PLC), pedicle, vertebral arch, transverse process, and articular process were erased in this phase to reduce computational efforts. After masking and model generation, the STL model of cement and vertebrae was exported to preprocessing software 3-Matic (Materialise NV, Harislee, Belgium) to generate mesh. According to Anitha et al. [18], thoracolumbar vertebra MDCT-FEA is acceptable for meshing with sensitivity errors decreasing to less than 10%. After the validation of meshing quality sensitivity on three random models within criteria (Figure 2), the volume mesh size of this study was set to a maximum 2 mm for both vertebrae and cement, and the overall volume mesh element type was set as tetrahedral C3D10.

The HU to element mechanical property conversion equation is listed in Table 2. The conversion of HU to apparent density (*ρ*, g/cm^3^) was performed according to previous FEA literature [19, 20]. The shift from elastic to postyield mechanical behavior of bone and cement was defined as bilinear isotropic hardening. Elastic modulus (*E*, MPa) was converted from apparent density according to Keller [21], and yield stress (*S*, MPa) was obtained from apparent density according to Morgan and Keveany [22]. The postyield modulus (*E*_py_, MPa) of the bilinear isotropic hardening model was set as 5% element elastic modulus [22]. Although the retrospective study was unable to collect an adequate number of quantitative computed tomography (QCT) scanned DICOM files that were in line with the calibration phantom, some phantom-less heterogeneous FEA suggested that with consistent scanner and scanning parameter, the mechanical results were identical with phantom calibrated one [23, 24]. The regression test in our study only requires accuracy of relative bone mechanics (the difference of mechanical properties between different vertebrae samples), and our DICOM data was obtained from consistent CT scanner with consistent parameters throughout the scan, such as KVP, X-ray tube current, reconstruction kernel, and pixel size. This was sufficient to run the regression and other test in our study.

The article "A Three-Dimensional Cement Quantification Method for Decision Prediction of Vertebral Recompression after Vertebroplasty" was retracted in 2023. Reasons: signs of a paper mill; suspected computer-generated content; unreliable results or conclusions; concerns about the data.

Moreover, this study also examined the mechanical behavior changes between 4 different homogeneous cement types. The elastic-perfect plastic model was assigned for cement. Cement strength and Young's modulus were adopted from literature in Table 3. The volume mesh file and material-to-element cross-reference file were fed to ANSYS workbench 19.0 (Ansys, Pennsylvania, USA).

### 2.3. Boundary Conditions and Convergence

Single vertebral uniaxial compression has been adopted in many studies, both in FEA and in vitro biomechanical tests [30–32]. A displacement load was applied to the upper endplate, as shown in Figure 1, to simulate uniaxial compression in a direction vertical to the lower endplate [33], and no degree of freedom was constrained. The step controls were defined by substeps. And the initial substeps were set as 30. The maximum substeps were set at 100. A fixed support was assigned at the lower endplate for complete constraint, and the reaction force of the fixed lower endplate was recorded while the displacement of the upper endplate continues (Figure 1). The failure load was defined as the resultant axial reaction force at compressive displacement of cranial endplate equal to 1.9% of minimum distance of two endplates [34], and stiffness was estimated as the slope of the linear range in force-displacement curves. The working environment was Ansys Mechanical APDL (ANSYS® Academic Research, Release 19.0, Pennsylvania, USA).

### 2.4. Quantification of Cement Distribution

1. Quantification of cement distribution extensiveness

To quantify the overall cement distribution, this study developed a stand-alone parameter called the distribution number (DN), which is independent of the cement volume (CV) and the cement volume fraction (VF%). Briefly, the 3D reconstructed vertebrae and cement cloud were divided into 27 portions (cubes) in three anatomic planes according to the vertebral anatomical structure by 6 splitting surfaces (Figure 3). Two coronal splitting surfaces were parallel to the spinous process, which were located on intersection of pedicles and vertebral foramen. Two sagittal splitting surfaces were placed in third of coronal splitting surfaces. The axial splitting surfaces were placed in third of vertebral front and posterior heights. The number of cement-occupied cubes was noted as the overall distribution number (oDN). To prevent invalid occupation in cubes, cement contact with three or more cube walls or cortical bone is certified as cement occupation within the cube.

(2) Quantification of endplate contact

The number of cement cubes touched the endplate was defined as the overall endplate contact number (oEP), which was a distribution parameter for subsequent regression analysis with failure load and stiffness, respectively.

(3) Definition of intravertebral regions

To explore the effect of cement distribution in different intravertebral regions, 27 cubes were classified as frontier column, middle column, and posterior column in the coronal direction (Figure 3(b)). In the transverse direction, 27 cubes were classified as superior transverse, middle transverse, and inferior transverse (Figure 3(c)). In each region of vertebrae, the regional distribution number (rDN), regional endplate contact number (rEP), regional volume fraction (rVF%), and regional cement volume (rCV) were noted. Finally, the linear regression *R*^2^ of CV, VF%, DN, and EP on the failure load and stiffness was calculated. The comparison of *R*^2^ showed that dominant factors affect augmentation.

The article "A Three-Dimensional Cement Quantification Method for Decision Prediction of Vertebral Recompression after Vertebroplasty" was retracted in 2023. Reasons: signs of a paper mill; suspected computer-generated content; unreliable results or conclusions; concerns about the data.

### 2.5. Statistical Analysis

*t*-tests and Wilcoxon rank sum tests were used to verify the differences in parameters between the PKP and PVP groups. The difference in failure load and stiffness between different types of cement was tested by the Wilcoxon rank sum test. The difference in the average was tested by a *t*-test (*n* = 51). Linear regression analysis was conducted to explore the possible relationship between multiple independent and dependent parameters, thus generating *R*^2^.

## 3. Results

### 3.1. Cement Distribution Quantification in PVP and PKP

The comparison of variables in the PVP and PKP groups is presented in Table 4. There was no significant difference in cement volume between PVP and PKP (*P* = 0.29). In addition, all independent variables (distribution parameter) and dependent variables exhibited significant differences between the two groups. The vertebral volume of the PKP group was significantly larger (34039.56 ± 13716.6 mm^3^) than that of the PVP group (25001.29 ± 5755.99 mm^3^), so it is reasonable that the PVP group exhibited a significantly larger oVF% than the PKP group.

The oEP was also significantly larger in the PVP group. For PKP, the cancellous bone tamped by the inflated balloon might be denser and harder to penetrate by PMMA, thus decreasing the value of oDN and oEP. The contrast figures of typical cement morphology in PVP and PKP groups are in Figure S4. Except for the CPC group, the failure load and stiffness of the PVP group were significantly higher than those of the PKP group (Table 4). Since there was a significant difference between the PKP and PVP groups in terms of independent variables (distribution parameter), predicted vertebral failure load, and stiffness, the subsequent regression analysis and Wilcoxon rank sum test were conducted for pooled data with PVP or PKP adjusted.

The article "A Three-Dimensional Cement Quantification Method for Decision Prediction of Vertebral Recompression after Vertebroplasty" was retracted in 2023. Reasons: signs of a paper mill; suspected computer-generated content; unreliable results or conclusions; concerns about the data.

Data were assessed by the Wilcoxon rank sum test; no significant mechanical difference was found between different groups of PMMA cement. The calcium phosphate cement group had significant lower failure load and stiffness than any PMMA cement group. 0.010 <  ^∗^*P* < 0.050 and ^∗∗^*P* < 0.010.

The mean oCV, oVF, oDN, and oEP for all vertebrae (pooled data) were 6259.6 ± 1653.88 mL, 23.13 ± 8.15%, 18.92 ± 3.43, and 4.18 ± 3.23, respectively. The predicted failure load of augmented vertebrae with four different types of cement was A: 2466.8 ± 1151.1 N, B: 2642.7 ± 1299.3 N, C: 2760.9 ± 1418.4 N, and D: 1986.19 ± 743.69 N, respectively. The predicted stiffness of augmented vertebrae with four different types of cement was A: 8587.5 ± 4958.7 N/mm, B: 9451.5 ± 5765 N/mm, C : 10010 ± 6277.9 N/mm, and D: 6597.28 ± 3175.08 N/mm, respectively. Different cement types had no significant impact on the predicted failure load and stiffness of augmented vertebrae except cement type D (calcium phosphate cement) in the Wilcoxon rank sum test (Figure 4).

### 3.2. Correlation of Overall Distribution Parameters with Strength and Stiffness

The linear regression analysis of vertebrae with cement type B is presented in Figure 5, and the corresponding analysis of the other three types of cement is available in the Supplementary materials (Table S1). The oDN exhibited a highest correlation with the failure load (*R*^2^ = 0.729); thus, this parameter had potential to be utilized as a postoperative fracture rack predictor. The lower oDN could be a sign of augmented vertebrae endanger by vertebral recompression even refracture. The oEP was most correlated with stiffness (*R*^2^ = 0.684) in this study (Figure 5(f)), indicating that cement-endplate contact could strongly affect augmented vertebrae stiffening. oCV and oVF% with determination coefficients of *R*^2^ = 0.4 and *R*^2^ = 0.286, respectively, indicating the oDN and oEP were better parameter for postoperative evaluation and prediction. No obvious collinearity was found between these overall distribution parameters and volumetric parameters after diagnosis (Figure 6). This statistically proves that oDN and oEP are independent of oCV and oVF%.

The article "A Three-Dimensional Cement Quantification Method for Decision Prediction of Vertebral Recompression after Vertebroplasty" was retracted in 2023. Reasons: signs of a paper mill; suspected computer-generated content; unreliable results or conclusions; concerns about the data.

### 3.3. Correlation of Regional Parameters with Strength and Stiffness

The linear regression test for regional independent variables in coronal planes with vertebral failure load with cement type B is presented in Figure 7(a). The front and middle column rDNs exhibited identical determination coefficients on failure load (*R*^2^ = 0.508 for front column and *R*^2^ = 0.49 for middle column). *R*^2^ of rEP on failure load was close between front and middle columns. A lower correlation was found between posterior column rDN and failure load (*R*^2^ = 0.206). Corresponding analyses of the other three types of cement are available in the Supplementary materials (Figures S1a, S2a, S3a). In terms of stiffness, rEP in the front column dominated vertebral stiffness changing, with *R*^2^ = 0.59 (Figure 7(b)).

For transverse planes, with cement type B, cement in the superior and inferior transverse planes produced a similar influence on the failure load when endplate contact occurred (Figure 7(c)). The rEP correlation on stiffness was highest (*R*^2^ = 0.421) in the inferior transverse (Figure 7(d)). Corresponding analyses of the other three types of cement are available in the Supplementary materials (Figures S1c, S1d, S2c, S2d, S3c, S3d). All regressions of regional variables on failure load and stiffness were significant (*P* < 0.05).

## 4. Discussion

Many common complications are caused by vertebra mechanical failure after vertebroplasty. Appropriate parameters should be proposed to describe the augmented vertebral mechanics. In this study, the intravertebral space was divided into 27 cubes, with a consistent quantification method, and cement distribution was parameterized as overall distribution number (oDN) and overall endplate contact number (oEP). Overall cement volume (oCV) and overall cement volume fraction (oVF%) were also determined. Additionally, the distribution parameters in three transverse (superior, midtransverse, and inferior) and three coronal (front, middle, and post) regions were noted as regional distribution number (rDN) and regional endplate contact number (rEP). The predictive value of these parameters was assessed by their correlation with cemented vertebral mechanics. This analysis was helpful in selection of proper parameters during postsurgical decision prediction process.

### 4.1. Correlation of Distribution Parameters and Mechanical Properties

To quantify cement morphology inside vertebrae, it was intuitive to divide the vertebrae into 27 cubes in three dimensions according to patient-specific vertebral anatomy. The method can be easily adopted to risk parameter evaluation before postsurgical decision-making process, like VAS score, kyphotic restoration, and vertebral height restoration, thus increase accuracy on decision-making process of revision surgery necessity. This kind of vertebral dividing method had been adopted by some recent vertebral bone mineral heterogeneity studies [35, 36].

The article "A Three-Dimensional Cement Quantification Method for Decision Prediction of Vertebral Recompression after Vertebroplasty" was retracted in 2023. Reasons: signs of a paper mill; suspected computer-generated content; unreliable results or conclusions; concerns about the data.

The results of the current study indicate that there was a strong positive correlation (*R*^2^ = 0.729) between oDN and the failure load (Figure 5(a)). To the authors' understanding, the oDN assesses the extensiveness of space occupied by cement and the even distribution of cement mechanical support. Multiple clinical studies had noted that interdigitated cement distribution instead of lump distribution can significantly decrease the chances of refracture [6, 7], and some research had emphasized that refracture of the augmented level may be due to uneven loading, which is initiated by the uneven distribution of cement [11, 12]. With more extensive cement distribution (higher oDN), the mechanical support of cement was typically even, and less intravertebral space remained unsupported. The oDN in this study could effectively quantify this extensiveness. The high *R*^2^ of oDN on failure load (*R*^2^ = 0.729) made this parameter available for vertebral recompression prediction postoperatively. The lower value of oDN indicated more risk for augmented vertebrae to fail. The oEP was regarded as quantified parameter of endplate contact, and it was correlated with vertebral stiffness (*R*^2^ = 0.684), and the *R*^2^ was the highest of all the variables (Figure 5(f)). Considering that the vertebral stiffness was correlated with adjacent new vertebral fracture [37, 38], the oEP could be utilized as predictor of new adjacent segment vertebral fracture postoperatively. Preoperatively, low oEP cement insert strategy in severe osteoporosis patients could prevent new adjacent segment vertebral fracture.

CV and VF% have been investigated as cement distribution parameters, but whether these factors can dominate the mechanical behavior of cemented vertebrae remains conflicted [9]. oCV and oVF% were compared with oDN and oEP, and the oVF% and oCV obtained relatively low *R*^2^ values for the predicted failure load and stiffness, which indicates that the mechanical properties of augmented vertebrae are not directly affected by VF% or CV (Figures 5(c), 5(d), 5(g), and 5(h)). The reason of that was the different dispersion resistances of various BMDs inside vertebrae can largely impact the final cement morphology for the same amount of CV or VF% [39]. Thus, the CV and VF% are inconsistent and unreliable scales to validate augmentation, and these parameters can be confounding for postsurgical decision-making. Different cement modulus cannot significantly decrease stiffness (Figure 4(b)) in our study.

The article "A Three-Dimensional Cement Quantification Method for Decision Prediction of Vertebral Recompression after Vertebroplasty" was retracted in 2023. Reasons: signs of a paper mill; suspected computer-generated content; unreliable results or conclusions; concerns about the data.

### 4.2. Mechanical Differences between PVP and PKP

Grouping information for PVP and PKP was collected along with DICOM from clinic in this study. No significant difference in oCV was found between the two groups, but the oDN, oEP, and mechanics all exhibited significant differences between the PVP and PKP groups.

The significant difference in oDN between the PVP and PKP groups may be due to the cancellous bone tamped by inflated balloons in the PKP groups, which can make cancellous bone denser and harder to penetrate by PMMA. The lump distribution pattern exhibited a lower oDN in this study, and PVP with interdigitated distribution [14, 40] could achieve a significantly increased oDN. A similar situation was observed for oEP between PVP and PKP groups, and more retention of the cancellous structure in PVP makes it easier for cement to disperse to the endplate [14, 41]. Compared with that of the PKP group, the oVF% in the PVP group was significantly higher, and it is mainly because the frontier vertebral height is generally higher after inflation of the balloon in PKP than in the PVP group in many studies [40, 41], which could cause the vertebral volume of the PKP group to increase during the masking procedure (Figure 1). As quantified by the cement distribution in this study, oDN and oEP were both significantly higher in the PVP group, indicating that the cement dispersed better in the PVP group.

The predicted failure load was significantly higher in the PVP group than in the PKP group, which corresponds to previous studies [40, 41]. The PKP group exhibited greater refracture incidence or loss of frontier height, and different cement distribution patterns were key factors according to previous studies, which corresponds with the results of this study. Thus, differentiation of PVP and PKP technique is crucial in postsurgical evaluation process because of significant lower failure load in the PKP group. In a similar situation regarding stiffness, the more interdigitated distribution in PVP increases the oDN and strength, while simultaneously increasing the oEP. The *R*^2^ of oEP on stiffness (*R*^2^ = 0.684) suggested that a higher oEP indicates greater stiffness in the PVP group (Table 4). Corresponding to previous clinical research [7, 41], the “stress-riser” effect occurring in PVP was more intense than that in PKP, leading to more adjacent vertebral compression.

The article "A Three-Dimensional Cement Quantification Method for Decision Prediction of Vertebral Recompression after Vertebroplasty" was retracted in 2023. Reasons: signs of a paper mill; suspected computer-generated content; unreliable results or conclusions; concerns about the data.

### 4.3. Distribution in Different Regions of Intravertebral Space

Different *R*^2^ for rDN and rEP on failure load across three columns reflected the load bearing mechanism of vertebrae (Figure 7(a)). The result was not only helpful for postsurgical evaluation and decision-making, but also beneficial for injection technique such as needle placement and needle movement. The three-column theory [42] indicated that the front column bears most of the vertebral axial load, and the front column in the three-column theory is similar to the front and middle columns of the vertebrae in this study, which were correlated with the failure load. This conclusion was consistent with a previous X-ray retrospective study: a greater cement distribution in the middle column was a protective factor against repeat collapse after surgery [8]. Moreover, endplate contact in the front column can aggressively affect vertebral stiffness (Figure 7(b)). To prevent adjacent vertebral fracture, the rEP in this region should be controlled within a reasonable range, and the overly high rEP in this region can be an alert for newly adjacent segment fracture in postsurgical inspection. The postcolumn distribution in this study barely shows any correlation with failure load or stiffness; however, it is not the indication that the cement dispersion in this region is unimportant. On the contrary, it has been reported that the presence of a basivertebral foramen indicates weakness of vertebral load bearing and could lead to the superior endplate failure and burst fracture [43]; therefore, the augmentation of postcolumn region cannot be ignored. In terms of different transverse regions (Figure 7(d)), rEP in the superior and inferior transverse exhibits similar and strong influence on stiffness. Gustafson et al. [44] reported that when a large compressive strain develops in near superior and inferior endplate regions when experiencing axial compression, the cement-endplate contact in both regions can ease the strain, thus improving the stiffness of the augmented vertebrae.

There are some drawbacks in this study. First, the sample size was limited by the number of patients, and the patients' CT data after vertebroplasty were difficult to obtain because of the instant pain reduction after this type of surgery, and patients tend to not return to clinic and undergo the CT inspection. Second, phantom CT calibration requires QCT scans; unfortunately, this retrospective study was unable to collect an adequate number of QCT scanned DICOM files containing the calibration phantom. With that said, the DICOM data were obtained from a consistent CT scanner, with consistent parameters throughout the scan, such as KVP, X-ray tube current, pixel size, and reconstruction kernel. Thus, the predicted mechanical differences between vertebrae are reliable, and therefore sufficient to calculate the *R*^2^ of cement distribution with vertebral mechanical properties.

The article "A Three-Dimensional Cement Quantification Method for Decision Prediction of Vertebral Recompression after Vertebroplasty" was retracted in 2023. Reasons: signs of a paper mill; suspected computer-generated content; unreliable results or conclusions; concerns about the data.

### 4.4. Further Application of Proposed Methods and Parameters

The proposed parameters, oDN, oEP, and rEP in front column, are well correlated with vertebral mechanics, and the combination of these parameter with IoHT (Internet of Health Things) system is promising (Figure 8). For patients performed vertebroplasty, their postoperative CT images stored in PACS (picture archiving and communication system) are analyzed, and generate diagnostic parameters by proposed methods. These parameters can be extracted from postoperative CT image by IoHT-based image recognition system [45–48], which can be done by local or cloud GPU (Graphics Processing Unit) without the need for specific hardware and user knowledge [49–51]. In some recent research, deep learning algorithm, CNN (Convolutional Neural Networks), and other techniques have been adopted to medical image process [52–55], and some algorithm is developed specifically for CT image recognition [56]. This kind of solution can be adopted to bone cement automatic parametrization. After oDN and oEP are extracted from image recognition algorithm, these parameters can be inputted into specific empirical formula on IoHT to generate risk indicator as auxiliary diagnose. Thus, medical specialist can propose a low latency and accurate diagnose for necessity of revision surgery. Meanwhile, the proposed parameters can also be used preoperatively to help surgeons to reduce the risk of cement leakage during the injection process. On the other hand, lower oEP in severe osteoporosis patients can prevent new adjacent segment vertebral fracture.

## 5. Conclusion

Three-dimensional cemented vertebral models were reconstructed based on MDCT data. By dividing the intravertebral space into 27 sections (cubes), a stand-alone method was developed to quantify intravertebral cement morphology. Different *R*^2^ values indicated that the extensive distribution of intravertebral cement (oDN) played an important role in augmented vertebral mechanical properties. The oDN and oEP were most correlated with the failure load and stiffness, respectively. Regionally, rDN in the front column and inferior transverse exhibited significant correlation with mechanical behavior. Proposed parameters have the potential to be used as a postoperative evaluation scale thus improving the quality of clinical decision-making, in this way to increase life quality of older people, reducing the public health pressure.

The article "A Three-Dimensional Cement Quantification Method for Decision Prediction of Vertebral Recompression after Vertebroplasty" was retracted in 2023. Reasons: signs of a paper mill; suspected computer-generated content; unreliable results or conclusions; concerns about the data.

## Figures and Tables

**Figure 1:** Overall flow chart of the imaging process and postvertebroplasty FEA model development. The boundary condition is imposed in step 5, blue arrows represent displacement compression, and red triangles represent fixation. Displacement was set at increments of 0.033 mm.

**Figure 2:** FEA mesh sensitivity validation. The rate of difference in mesh sizes was calculated by the mechanical difference of a 0.5 mm mesh size model.

**Figure 3:** oDN quantification method: vertebrae and cement were anatomically divided into 27 portions. The red box indicates the alignment position of 6 splitting surfaces in three anatomical surfaces. Blue lines represent region division. Fr: front column; Mid: middle column; Po: postcolumn; Sup: superior transverse; Mid-T: middle transverse; Inf: inferior transverse. The number of cement-occupied cubes was noted as oDN, and the number of cement cubes touching the endplate was noted as oEP. (a) Transverse plane; (b) sagittal plane; (c) coronal plane; (d) overview in three dimensions.

**Figure 4:** Mechanical properties of vertebrae with different types of cement. (a) Failure load in four types of cement and (b) stiffness in four types of cement.

**Figure 5:** Linear regression analysis of distributional parameters on predicted (a–d) failure load and (e–h) stiffness; all regressions are significant (*P* < 0.05).

**Figure 6:** Collinearity diagnosis of overall independent variables. oDN and oEP are independent of oCV and oVF%.

**Figure 7:** Determination coefficient of regional variables on failure load and stiffness of cement type B. (a) *R*^2^ of different regional variables on failure load in three coronal regions, (b) *R*^2^ of different regional variables on stiffness in three coronal regions, (c) *R*^2^ of different regional variables on failure load in three transverse regions, and (d) *R*^2^ of different regional variables on stiffness in three transverse regions.

**Figure 8:** Application of patient-specific vertebroplasty parameters for postoperative decision-making process.

**Table 1:** Statistical review of patients' augmented levels.

PVP (*n* = 24)		PKP (*n* = 27)	
Levels	Numbers	Levels	Numbers
T10	0	T10	1
T11	3	T11	6
T12	9	T12	7
L1	4	L1	6
L2	5	L2	4
L3	2	L3	0
L4	1	L4	3

**Table 2:** Material property relations adopted from the literature.

Parameters	Mathematical relationship	References
Apparent density (g/cm^3^)	*ρ* = 0.001 × (1.3465 + 0.945HU)	Mazlan et al. [19] [20]
Elastic modulus (MPa)	*E* = 757 × *ρ*^1.94^	Keller [21]
Yield stress (MPa)	*S* = 21.7 × *ρ*^1.52^	Morgan and Keaveny [22]
Postyield modulus (MPa)	*E*_py_ = 0.05 × 757 × *ρ*^1.94^	Morgan and Keaveny [22]
Poisson ratio	0.3	

The article "A Three-Dimensional Cement Quantification Method for Decision Prediction of Vertebral Recompression after Vertebroplasty" was retracted in 2023. Reasons: signs of a paper mill; suspected computer-generated content; unreliable results or conclusions; concerns about the data.

**Table 3:** Material properties of homogeneous bilinear bone cements adopted from the literature.

Types of cement	Young's modulus (GPa)	Strength (MPa)	References
Cement type A (low modulus PMMA)	1.5	85	Robo et al. [25]
Cement type B (medium modulus PMMA)	2.5	90	Wekwejt et al. [26]
Cement type C (high modulus PMMA)	3.5	95	López et al. [27]
Cement type D (calcium phosphate cement)	0.5	10	Palmer et al. [28]; Liu et al. [29]

**Table 4:** Comparison of different variables between the PVP and PKP groups (mean ± SD).

Variables	PVP (*n* = 24)	PKP (*n* = 27)	*P* value
Distribution parameter (independent variables)			
Vertebral volume (mm^3^)	25001.29 ± 5755.99	34039.56 ± 13716.63	0.003
oCV (mm^3^)	6515 ± 1167	6032 ± 1985	0.290
oVF% (mm^3^/mm^3^ %)	26.79 ± 5.41	19.88 ± 8.87	0.002
oDN (-)	20 ± 3.49	17.96 ± 3.14	0.033
oEP (-)	5.42 ± 3.12	3.07 ± 2.96	0.009
Mechanical parameters (dependent variables)			
Failure load with cement A (N)	2791.9 ± 1198.3	2177.89 ± 1045.83	0.048
Stiffness with cement A (N/mm)	10467.11 ± 4859.22	6916.67 ± 4498.73	0.001
Failure load with cement B (N)	3026.73 ± 1345.37	2301.25 ± 1178.22	0.045
Stiffness with cement B (N/mm)	11643.87 ± 5594	7502.66 ± 5277.48	0.001
Failure load with cement C (N)	3200.55 ± 1493.49	2370.1 ± 1248.52	0.042
Stiffness with cement C (N/mm)	12370.57 ± 6030.68	7911.84 ± 5822.76	0.001
Failure load with cement D (N)	2157.28 ± 788.03	1834.1 ± 680.6	0.117
Stiffness with cement D (N/mm)	7875.3 ± 3245.27	5461.26 ± 2687.45	0.001

*P* values of independent variables are from independent sample *t*-tests because they are normally distributed. *P* values of predicted mechanical variables are from Wilcoxon rank sum tests.

## Data Availability

The datasets used and analyzed during the current study are available from the corresponding author on reasonable request.

## Supplementary Materials

Supplementary Materials The supplementary file includes regression results of different types of bone cement in FEA study. Table S1 shows determination coefficients of overall parameters on failure load and stiffness in four types of cement. Figure S1 shows determination coefficients of regional parameters on failure load and stiffness in cement type A. Figure S2 shows determination coefficients of regional parameters on failure load and stiffness in cement type C. Figure S3 shows determination coefficients of regional parameters on failure load and stiffness in cement type D. Figure S4 shows contrast of typical cement morphology in PVP and PKP groups.
